This article has been retracted.

# Psorinum Therapy in Treating Stomach, Gall Bladder, Pancreatic, and Liver Cancers: A Prospective Clinical Study

**DOI:** 10.1155/2011/724743

**Published:** 2010-12-08

**Authors:** Aradeep Chatterjee, Jaydip Biswas, Ashim Chatterjee, Sudin Bhattacharya, Bishnu Mukhopadhyay, Syamsundar Mandal

**Affiliations:** ^1^Critical Cancer Management Research Centre & Clinic, 381 S K Deb Road, West Bengal, Kolkata 700 048, India; ^2^Chittaranjan National Cancer Institute, Kolkata 700 026, India; ^3^National Institute of Technology, Durgapur 713209, India

## Abstract

We prospectively studied the clinical efficacy of an alternative cancer treatment “Psorinum Therapy” in treating stomach, gall bladder, pancreatic and liver cancers. Our study was observational, open level and single arm. The participants' eligibility criteria included histopathology/cytopathology confirmation of malignancy, inoperable tumor, and no prior chemotherapy or radiation therapy. The primary outcome measures of the study were (i) to assess the radiological tumor response (ii) to find out how many participants survived at least 1 year, 2 years, 3 years, 4 years and finally 5 years after the beginning of the study considering each type of cancer. Psorinum-6x was administered orally to all the participants up to 0.02 ml/Kg body weight as a single dose in empty stomach per day for 2 years along with allopathic and homeopathic supportive cares. 158 participants (42 of stomach, 40 of gall bladder, 44 of pancreatic, 32 of liver) were included in the final analysis of the study. Complete tumor response occurred in 28 (17.72%) cases and partial tumor response occurred in 56 (35.44%) cases. Double-blind randomized controlled clinical trial should be conducted for further scientific exploration of this alternative cancer treatment.

## 1. Introduction

Although, great advances have been made in the treatment of some forms of cancer and new advances in surgery, radiotherapy, and chemotherapy leading to an increase in cure rates have been achieved, such interventions are often too much expensive and beyond the reach of many cancer patients of the developing as well as of the developed countries [1–3]. In developing countries, majority of the cancer patients have inadequate access to the mainstream cancer treatments due to lack of proper medical infrastructures, skills, and above all limited financial resources [4, 5]. Some types of cancer (i.e., liver, gall bladder, pancreatic, and stomach) are still associated with poor prognosis to conventional cancer treatments [6–9]. Side effects of the chemotherapy and radiation therapy are also intolerable to many cancer patients [10–12]. In most of the situations, elderly cancer patients cannot be provided with conventional cancer treatments because of old age-related problems [13, 14]. As a result, alternative cancer treatments have become an important feature of oncology regardless of geographic region and they appear to exist in greater abundance through out the world. Many alternative cancer therapeutic modalities are now being practiced in India, and one of them which has gained significant popularity is called Psorinum Therapy [15–17]. The investigational anticancer drug used in this alternative cancer therapy is “Psorinum” which is derived from the sphere of homeopathy. The supportive treatments of Psorinum Therapy are adopted both from the spheres of allopathy and homeopathy. Psorinum is an alcoholic extract of the scabies, slough, and pus cells. According to the pre-clinical data, “Psorinum-6x” (“x” stands for decimal potency of homeopathy) activates different immune effector cells (e.g., T cells, and accessory cells like, macrophages, dendritic cells, and natural killer cells) which can trigger a complex antitumor immune response [18, 19]. In a rat model study, daily oral administration of Psorinum 6x at doses up to 0.5 ml/Kg body weight/day for 2 weeks resulted in no adverse side effect [19]. Published retrospective and prospective studies also support the efficacy of Psorinum Therapy in treating patients with various malignancies [20–28]. The prospective observational clinical trial, reported here, was conducted to evaluate the efficacy of the Psorinum Therapy in treating stomach, gall bladder, pancreatic, and liver cancers and to assess the side effects of the drug Psorinum if any [29]. 

## 2. Materials and Methods

### 2.1. Settings

The study was conducted by the Critical Cancer Management Research Centre and Clinic (CCMRCC) situated in Kolkata of West Bengal, India. The study started from June 2001 and completed in July 2009. The study protocol was approved by the Institutional Review Board (IRB approval Number: 2001–05) of the CCMRCC in conformity with the World Medical Association (WMA) declaration of Helsinki and it is subsequent amendments and the ethical guidelines of the Indian Council of Medical Research (ICMR) for the biomedical research on human participants.

### 2.2. Study Design

The study was prospective, observational, open level, and single arm. 

### 2.3. Inclusion and Exclusion Criteria

Only the patients of confirmed malignancy (by histopathological examination of endoscopic biopsy, cytopathological exam of CT guided FNAC) involving stomach, gall bladder, pancreatic, and liver cancers of both sexes were enrolled. The participants' eligibility criteria included (i) histopathology/cytopathology confirmation of malignancy, (ii) inoperable tumors, and (iii) no prior chemotherapy or radiation therapy. The lower age limit was 18 years and there was no upper age limit for the eligibility. Patients who were unable to understand English, Hindi, or Bengali or resided outside India were excluded from the study. The patients who reported the cancer centre from the period of June 2001 to November 2003 and fulfilled the eligibility criteria were recruited. Written informed signed consent was taken from each patient before starting the study.

### 2.4. Intervention

Psorinum-6x was administered orally to all the participants up to 0.02 ml/Kg body weight as a single dose in empty stomach per day for complete course duration of 2 years.

### 2.5. Supportive Treatments

In this study, the supportive cares were taken both from the spheres of allopathy and homeopathy. Supportive cares for control of infection, pain, electrolytic balance, bleeding, nutritional deficiencies were taken, and blood transfusion, abdominal or plural paracentesis, analgesic, bronchodilator, stenting of the hepato-pancreato-biliary system, and bypass were done as and when required to improve the survival and the quality of life of the participants. The frequently used homeopathic medicines for the purpose of the supportive cares were *Chelidonium majus, Carduus marianus, Baryta carbonica, Conium maculatum*, *Carbo animalis, Bryonia alba, Medorrhinum, Thuja occidentalis, Cholesterinum, and Lycopodium clavatum* (Table 1). Less frequently used homeopathic medicines for the purpose of the supportive cares were mother tincture of the *Berberis vulgaris*, mother tincture of the *Calendula officinalis*, mother tincture of the *Hamamelis virginiana*, mother tincture of the *Symphytum officianale*, mother tincture of the *Syzygium jambolanum*, *Gelsemium* 200c, *Cantharides* 200c, *Sulphur* 200c, *Arsenicum album *200c, and *Causticum* 200c.

### 2.6. Outcome Measures

Primary outcome measures of the study were (i) to assess the radiological tumor response and (ii) to find out in each type of cancer how many participants survived at least 1 year, 2 years, 3 years, 4 years, and finally, after 5 years since the beginning of the study. To assess the radiological tumor response, CT Scans were done at the beginning of the study, repeated every 3–6 months during the 1st year of the study and repeated every 6–8 months during the next 2 years of the study. Radiological tumor response was defined by Response Evaluation Criteria in Solid Tumors (RECIST). A complete response was defined as complete disappearance of all targeted lesions without disease progression or any new lesion, and a partial response was defined as at least 30% regression in the sum of the longest diameter of the targeted lesions as reference to the baseline sum LD without disease progression or any new lesion. To assess the survival, the investigators followed up the participants via personal meetings, phone calls, and mails at least for 5 years (where applicable) after the study began. Secondary outcome measure of the study was to assess the side effects of the Psorinum. The investigators asked the participants and also examined them clinically to assess if they had any side effect. Apart from these, participants were also followed up to know if they were taking any other conventional or investigational cancer treatments.

## 3. Results

10 (5.95%) participants were dropped out from the study as they opted for conventional cancer treatments, among them 4 of stomach, 2 of gall bladder, 3 of pancreatic, and 1 of liver cancers. 158 participants (42 of stomach, 40 of gall bladder, 44 of pancreatic, and 32 of liver) were included in the final analysis at the end of the study. In these participants, the diagnosis of malignancies was confirmed by histopathological examination of endoscopic biopsies and cytopathological examination of CT-guided FNAC. In case of stomach, gall bladder, and pancreatic cancers, the histology type was adenocarcinoma, and in case of liver cancer the histology type was hepato cellular carcinoma (HCC). Among the 158 participants, 84 (53.16%) were male and 74 (46.84%) were female. According to the AJCC TNM staging system, 39 (24.68%) were diagnosed at stage-III, and 112 (70.89%) were diagnosed at stage-IV. The participants' Karnofsky status was between 40–70%, and Eastern Cooperative Oncology Group (ECOG) status was between 2-3. Among the 39 participants (24.68%) who were diagnosed at stage-III, 13 (33.33%) had complete response and 16 (41.03%) had radiological partial response. Among the 112 (70.89%) participants who were diagnosed at stage-IV, 12 (10.71%) had radiological complete response and 38 (33.93%) had radiological partial response (Tables 2 and 3, Figures 1, 2, and 3). In this study, no adverse side effects were observed from the drug Psorinum. However, very few patients reported to have mild oral irritation and skin itching which were successfully controlled by the supportive cares. Psorinum Therapy was also effective in improving the disease symptoms and the quality of life of the participants. At least 60% participants of stage-III and at least 45% participants of stage-IV reported that the therapy was effective in reducing their cancer-related pain, cough, dysponea, nausea and vomiting, fatigue, constipation and improving appetite, and weakness. These were also confirmed after examining the participants clinically. Improvements were also observed in the lab investigations like Complete Blood Count (CBC), Liver Function Test (LFT), Kidney function test, AFP level, and CA 19.9. These lab investigations were done as a part of their routine clinical check ups. Among the 158 participants, 98 (62.03%) were aged 65 years or more. Better outcomes were observed among the participants below 65 years of age than the participants who were over the age of 65. The outcomes did not vary significantly while considering gender. Figures 4(a) and 4(b) show complete tumor response in one stomach and one gall bladder cancer patients, respectively, who were treated through Psorinum Therapy.

## 4. Discussion and Conclusion

Many studies were published on the role of complementary and alternative medicines in treating cancer patients. Some studies support the CAM therapies to be beneficial for palliative cancer cares [30–35]. However, very few of the published reports support their efficacy with regard to the primary care of cancer. According to our knowledge, the clinical study, reported here, is the only prospective study that intrigued a fair number of complete and partial tumor responses along with impressive survival outcomes in treating patients with stomach, gall bladder, pancreatic, and liver cancers through psorinum therapy. Previously, interviews were conducted on 300 biopsy-proved cancer patients of Psorinum Therapy. The primary purpose of the study was to ascertain the patients' and/or their caregivers' view on this CAM therapy. The survey showed the patients had tried Psorinum Therapy mainly due to no other available treatment options, financial constraints, frustration with the conventional cancer treatments, and belief in the efficacy of the Psorinum Therapy. According to the survey, among the 300 cancer patients, 195 (65%) had consulted their oncologists before trying the therapy [17]. This therapy can be easily replicated by other practitioners in different clinical centers due to the following advantages.

The reagent to prepare the drug Psorinum is available. The specific dosing and the medicinal power are established. The medicine administration technique is easy as it can be taken orally. 

The supportive treatments are adopted from the allopathic streams. The supportive treatments with homeopathic medicines are done by specific ailment versus specific medicine concept instead of the concept of specific patient versus specific medicine, making the homeopathic supportive cares easier to replicate. In a nutshell, we should remember that, 158 participants of histopathology or cytopathology confirmed stomach, gall bladder, pancreatic, and liver cancers were included in the final analysis at the end of the study. According to the AJCC TNM staging system, 39 (24.68%) were diagnosed at stage-III and 112 (70.89%) were diagnosed at stage-IV. The participants Karnofsky status was between 30–60% and ECOGstatus was between 2-3. The participants received the drug Psorinum along with allopathic and homeopathic supportive treatments without trying conventional or any other investigational cancer treatments. According to the RECIST criteria, radiological complete response occurred in 28 (17.72%) and partial response occurred in 56 (35.44%) participants. The limitation of this study is that it did not have any placebo or treatment control arm; therefore, it cannot be concluded that Psorinum Therapy is effective in improving the survival and the quality of life of the participants due to the academic rigours of the scientific clinical trials. This study also cannot rule out the effects of the implemented allopathic and homeopathic supportive measures in the observed results. However, the results of the study showed a fair number of complete and partial tumor responses along with impressive survival outcomes in difficult to treat cancer types. Therefore, randomized double-blind clinical trial, detailed molecular, pharmacokinetics, and pharmacodynamics studies should be conducted for further scientific exploration of this alternative cancer treatment to determine if it can be integrated into the mainstream oncology.

## Figures and Tables

**Figure 1:** Distribution of partial and complete tumor response rates in different cancer types.

**Figure 2:** Lorenz Analysis: Distribution of tumor response in different cancer types.

**Figure 3:** Kaplan Meier survival analysis in different cancer types.

**Figure 4:** (a) Showing complete tumor response of a stomach cancer patient who underwent Psorinum Therapy. (b) Showing complete tumor response of a gall bladder cancer patient who underwent PsorinumTherapy.

**Table 1:** Details of the frequently used homeopathic medicines for the purpose of the supportive cares.

Name	Origin	Dosing	Power	Used to control ailments
(1) *Chelidonium majus *	Herb-*Chelidonium majus *	Up to 0.04 ml/Kg body weight/day orally	Mother tincture	(1) Abnormal liver functions (2) Dysponea
(2) *Carduus marianus *	Herb-*Carduus marianus *	Up to 0.04 ml/Kg body weight/day orally	Mother tincture	(1) Abnormal liver function (2) Cholestasis
(3) *Baryta carbonica *	Barium carbonate	Up to 0.02 ml/Kg body weight/day orally	200c	(1) Anaemia (2) Cancer-related pain
(4) *Conium maculatum *	Herb-*Conium maculatum *	Up to 0.02 ml/Kg body weight/day orally	200c	(1)Heart troubles (2) Abnormal blood pressure
(5) *Carbo animalis *	Animal charcoal	Up to 0.02 ml/Kg body weight/day orally	200c	(1) Cough (2) Constipation
(6) *Bryonia alba *	Herb-*Bryonia alba *	Up to 0.02 ml/Kg body weight/day orally	200c	(1) Dysponea (2) Cancer-related pain
(7) *Medorrhinum *	*Gonorrhoeal cocci*	Up to 0.02 ml/Kg body weight/day orally	200c	(1) Abnormal blood sugar (2) Cancer-related pain
(8) *Thuja occidentalis *	Herb-*Thuja occidentalis *	Up to 0.02 ml/Kg body weight/day orally	Mother tincture	(1) Abdominal distension (2) Electrolytic imbalance
(9) *Cholesterinum *	Cholesterine	Up to 0.02 ml/Kg body weight/day orally	200c	(1) Abnormal liver function (2) Cholestasis
(10) *Lycopodium clavatum *	Herb-*Lycopodium clavatum *	Up to 0.02 ml/Kg body weight/day orally	200c	(1) Abdominal distension (2) Cancer-related pain

c → Centesimal potency of homeopathy.

**Table 2:** TNM Staging, partial and complete tumor response in each cancer type.

Primary cancer types	No. of participants	TNM Staging of the participants		No. of patients: Complete tumor response occurred	No. of patients: Partial tumor response occurred
		Diagnosed at stage-II and stage-III	Diagnosed at stage-IV		
Stomach	42	11	31	6 (14.29%)	16 (38.1%)
G. Bladder	40	13	27	7 (17.5%)	17 (42.5%)
Pancreas	44	9	35	8 (18.18%)	13 (29.55%)
Liver	32	13	19	7 (21.87%)	10 (31.25%)

**Table 3:** Survival outcomes in each cancer type.

Primary organ affected	No. of Patients	Male	Female	Survived at least 1 year	Survived at least 2 years	Survived at least 3 years	Survived at least 4 years	Survived at least 5 years
Stomach	42	22	20	34	24	21	20	16 (38.1%)
G. Bladder	40	21	19	32	25	20	18	15 (37.5%)
Pancreas	44	24	20	34	28	27	21	17 (38.64%)
Liver	32	17	15	26	22	19	17	14 (43.75%)
